This article has been retracted.

# The Bicarbonate Transporter Is Essential for *Bacillus anthracis* Lethality

**DOI:** 10.1371/journal.ppat.1000210

**Published:** 2008-11-21

**Authors:** Adam C. Wilson, Magali Soyer, James A. Hoch, Marta Perego

**Affiliations:** The Scripps Research Institute, Department of Molecular and Experimental Medicine, Division of Cellular Biology, La Jolla, California, United States of America; Schepens Eye Research Institute, United States of America

## Abstract

In the pathogenic bacterium *Bacillus anthracis*, virulence requires induced expression of the anthrax toxin and capsule genes. Elevated CO_2_/bicarbonate levels, an indicator of the host environment, provide a signal ex vivo to increase expression of virulence factors, but the mechanism underlying induction and its relevance in vivo are unknown. We identified a previously uncharacterized ABC transporter (BAS2714-12) similar to bicarbonate transporters in photosynthetic cyanobacteria, which is essential to the bicarbonate induction of virulence gene expression. Deletion of the genes for the transporter abolished induction of toxin gene expression and strongly decreased the rate of bicarbonate uptake ex vivo, demonstrating that the BAS2714-12 locus encodes a bicarbonate ABC transporter. The bicarbonate transporter deletion strain was avirulent in the A/J mouse model of infection. Carbonic anhydrase inhibitors, which prevent the interconversion of CO_2_ and bicarbonate, significantly affected toxin expression only in the absence of bicarbonate or the bicarbonate transporter, suggesting that carbonic anhydrase activity is not essential to virulence factor induction and that bicarbonate, and not CO_2_, is the signal essential for virulence induction. The identification of this novel bicarbonate transporter essential to virulence of *B. anthracis* may be of relevance to other pathogens, such as *Streptococcus pyogenes*, *Escherichia coli*, *Borrelia burgdorferi*, and *Vibrio cholera* that regulate virulence factor expression in response to CO_2_/bicarbonate, and suggests it may be a target for antibacterial intervention.

## Author Summary

Hospital-acquired bacterial infections are a growing public health concern. The bacteria responsible for these infections are often resistant to multiple antibiotics, making the problem of nosocomial infections even more dramatic and the need for new antibacterial treatment more urgent. Bacteria rely on a variety of mechanisms in order to trigger an infection, but the first step must be the recognition of the host environment. In this work, we have identified the first component of a pathway that allows a bacterial pathogen, *Bacillus anthracis*, to recognize the environment in which to thrive during an infection, i.e. the blood of the host. The molecule sensed is bicarbonate, a critical component in the blood for maintaining its correct pH. Bicarbonate is essential to induce the virulence factors of *B. anthracis* and is most likely relevant in infections by other organisms such as *Streptococci*, *E. coli*, *Borrelia*, *Clostridium botulinum*, and *Vibrio cholera*. Our identification of the *B. anthracis* transporter responsible for the internalization of bicarbonate and the activation of virulence factor production provides a new target for new antibacterial intervention that could be effective on a variety of bacterial pathogens.

## Introduction

*Bacillus anthracis* is a Gram-positive, endospore-forming bacterium that is the etiological agent of anthrax. Anthrax is primarily a disease of grazing herbivores with human infections as the result of either direct contact with infected animal products or intentional dispersion of anthrax spores as a biological weapon. Anthrax can manifest as localized, cutaneous infections or as systemic infections resulting from spore inhalation, ingestion, or spread of cutaneous infections. While localized, cutaneous infections are curable, systemic infections are almost uniformly fatal with death occurring within days of initial infection [1].

Virulence in the mammalian host requires expression of both the anthrax toxin and the antiphagocytic capsule. The tripartite anthrax toxin is encoded by three non-contiguous genes, *lef*, *cya* and *pagA*, carried on the virulence plasmid pXO1 [2]. *lef* encodes Lethal Factor (LF), a zinc metalloprotease targeting host MAP-kinase signaling [3], *cya* encodes Edema Factor (EF), an adenylate cyclase that increases cellular cAMP levels [4], and *pagA* encodes Protective Antigen (PA), which forms a pore allowing entry of toxin components [5]. The antiphagocytic, poly-D-glutamic acid capsule, which is essential for bacterial dissemination in the host [6], is encoded by genes in the *cap* operon carried on virulence plasmid pXO2 [7],[8]. The regulatory protein AtxA, encoded by the *atxA* gene on pXO1, is required for the transcription of both the toxin genes and the capsule operon [9],[10]. Control of AtxA, in turn, is integrated into several metabolic regulatory circuits, including the sporulation phosphorelay through AbrB [11] and the phosphoenolpyruvate-dependent phosphotransferase system via regulated phosphorylation/dephosphorylation of histidine residues [12].

Many environmental cues influence the expression of *B. anthracis* virulence factors, one of the earliest identified being the effect of CO_2_/bicarbonate levels on capsule production and virulence [13]. Elevated CO_2_/bicarbonate levels are thought to serve as a signal of the mammalian host environment and a cue to induce expression of virulence factors. Incubation of *B. anthracis* in media supplemented with sodium bicarbonate and grown under elevated CO_2_ levels (above 5%) results in an approximately 10-fold increase in transcription of all three toxin genes [14] and a more than 20-fold increase in capsule operon transcription [15]. AtxA is required for CO_2_/bicarbonate induction of toxin and capsule genes, however, AtxA expression is unaffected by increased CO_2_/bicarbonate levels [16],[17]. The presence of additional CO_2_/bicarbonate regulatory components on the main chromosome is suggested by the observation that *pagA* transcription is induced by CO_2_/bicarbonate in a pXO1^−^ pXO2^−^ strain when *atxA* and *pagA* only are supplied on multicopy plasmids [18]. Additionally, an uncharacterized gene carried on pXO1 may also play a role in CO_2_/bicarbonate regulation of toxin expression [19]. Notwithstanding these indirect suggestions of more extensive regulation, additional CO_2_/bicarbonate regulatory components have yet to be directly identified.

Without a mechanistic basis for the CO_2_/bicarbonate regulation of virulence factor expression, our focus turned to identifying conserved responses to CO_2_/bicarbonate homeostasis and relating these pathways to *B. anthracis*. Study of CO_2_/bicarbonate metabolism is complicated by its labile nature, with CO_2_, H_2_CO_3_, HCO_3_^−^, and CO_3_^2−^ existing in equilibrium depending on pH, temperature, and partial pressure of CO_2_. Under typical biological conditions, CO_2_ generally diffuses across membranes; once inside the cell, carbonic anhydrases can actively interconvert CO_2_ and bicarbonate. On the other hand, bicarbonate is impermeable across lipid bilayers, and many cellular systems rely on dedicated transporters to import bicarbonate [20]. One of the best-studied bacterial bicarbonate transporters is the CmpABCD ABC transport system in the cyanobacterial species *Synechococcus* PCC 7942 (Figure 1) [21]. In this bacterium, elevated CO_2_ concentration around ribulose-1,5-bisphosphate carboxylase/oxygenase (Rubisco) is essential for efficient carbon fixation. *Synechococcus* uses this high affinity bicarbonate transporter to import and accumulate inorganic carbon (such as HCO_3_^−^), which can then be converted by carbonic anhydrase to CO_2_ in the presence of Rubisco in a specialized compartment called the carboxysome [22].

**Figure 1:** Schematic representation of the ABC-type transporters of bicarbonate in *Synechococcus*. The Substrate Binding Protein CmpA is presumably anchored to the periplasmic face of the cytoplasmic membrane via a lipid anchor attached to a conserved cystine at the end of a lipoprotein signal peptide [45]. The SBP domain is composed of two domains organized in a C-clamp shape [23]. In *Synechococcus*, a SBP domain is also present intracellularly at the carboxy terminal end of the CmpC ATPase subunit. The CmpC protein is absent in *B. anthracis* and in *S. pyogenes*. Also, in *S. pyogenes*, the SBP domain is fused at its C-terminal end to the CmpB-like permease domain.

Here we report the identification of an ABC transporter with similarity to the *Synechococcus* CmpABCD system that is essential to virulence in *B. anthracis*. Deletion of the genes for the transporter reduced bicarbonate uptake and eliminated toxin gene induction *ex vivo* in response to bicarbonate. More importantly, the strain lacking the transporter was avirulent in a mouse model of anthrax infection, demonstrating the importance of this pathway for recognition of the host environment and pathogenesis.

## Results

### Identification of a putative bicarbonate ABC transporter

Despite the recognized role of CO_2_/bicarbonate in toxin synthesis, the mechanism linking CO_2_/bicarbonate levels to toxin regulation and virulence of *B. anthracis* remains to be characterized. As a reverse genetic approach to identify components of the CO_2_/bicarbonate regulatory pathway, we searched the *B. anthracis* Sterne strain genome (GenBank: AE017225) for protein sequences similar to the products of the *cmpABCD* operon encoding the bicarbonate transporter of *Synechococcus elongatus* PCC 6301 (GenBank: AP008231). Unlike many ABC transporters, which are characterized largely based upon multisubunit organization including proteins with ABC-type ATP-binding domains in association with hydrophobic permease domains, identification of CmpABCD-like bicarbonate ABC transporters is aided by structural features of the substrate binding domain for bicarbonate and the highly similar nitrate transporters [23],[24].

A BLASTP search revealed similarity between components of CmpABCD system and the products of the BAS2714-12 and BAS4675-77 genes (Table 1). Both operons had yet to be characterized but appeared to encode components of ABC transporters. BAS2714 and BAS4676 encode ATP-binding proteins, BAS2713 and BAS4675 are predicted to encode substrate binding proteins, and BAS2712 and BAS4677 are likely transmembrane permease proteins. Unlike *cmpABCD*, which encodes two ATP-binding proteins (CmpC, also containing a CmpA-like substrate-binding protein, and CmpD) (Figure 1), the two *B. anthracis* loci encode only one single-domain ATP-binding protein (BAS2714 or BAS4676). A role in bicarbonate transport was suggested by the presence in the BAS2713 and BAS4675 proteins of a TauA domain (NCBI Accesion Number COG0715), a conserved element associated with periplasmic substrate binding components of ABC transporters specific for nitrate, sulfonate, or bicarbonate. Furthermore, a fold-recognition bioinformatic analysis by the FFAS03 server revealed a highly significant score (−60.5 to −64.8) between BAS2713 or BAS4675 and the bicarbonate (CmpA) and nitrate (NrtA) substrate binding protein, suggesting a structural and functional homology despite the limited sequence conservation. Based on similarity to the CmpABCD proteins and conserved features shared by bicarbonate transporters, the BAS2714-12 and BAS4675-77 systems appeared to be good candidates to function as a *B. anthracis* bicarbonate ABC transporter.

**Table 1:** Similarity analysis between the *B. anthracis* BAS2714-12 and BAS4675-77 transporter and the *Synechococcus* bicarbonate transporter CmpABCD.

	CmpC		CmpD		CmpA		CmpB	
**Gene**	BAS2714		BAS2714		BAS2713		BAS2712	
**P-value**	BAS4676		BAS4676		BAS4675		BAS4677	
**Identity**	5e-49	1e-43	6e-46	5e-37	.11	5e-06	7e-26	1e-09
**%**	40	38	40	34	23	25	31	25

P-value and percentage of identity were obtained using BlastP.

### Deletion of BAS2714-12 eliminates bicarbonate-induced toxin gene expression

To investigate the role of BAS2714-12 and BAS4675-77 in bicarbonate metabolism and virulence, *B. anthracis* 34F2 (pXO1^+^ pXO2^−^) derivative strains were generated containing a markerless deletion of the three genes annotated as BAS2714-12 or BAS4675-77. As described in the Experimental Procedures, using plasmid pAW091, a region from 97 nucleotides upstream of the translation start site of BAS2714 to 33 nucleotides upstream of the termination codon of BAS2712 was deleted. This completely eliminated the coding regions of BAS2714 and BAS2713 while leaving a small portion of the 3′ end of the BAS2712 coding sequence and the entire intergenic region between BAS2712 and BAS2711 intact so as to leave potential regulatory sequences controlling expression of the downstream gene, BAS2711.

Similarly, for the deletion of BAS4675-77, the integration of plasmid pAW093 resulted in the deletion of a region from 70 nucleotides downstream of the translation start site of BAS4675 to 52 nucleotides upstream of the termination codon of BAS4677. This completely eliminated the coding regions of BAS4676 while leaving a small portion of the 5′ end of the BAS4675 coding sequence and a small portion of the 3′ end of the BAS4677 coding sequence intact so as to leave potential regulatory sequences controlling expression of genes upstream and downstream of the operon.

Under all conditions tested, deletion of BAS2714-12 or BAS4675-77 had no significant effect on growth relative to the parental strain 34F2 (Figure 2 and data not shown).

**Figure 2:** Cell growth and virulence gene expression in *B. anthracis* 34F2 and 34F2ΔBAS2714-12 under various growth conditions. For β-galactoside assays, cells carrying a *pagA-lacZ* or *atxA-lacZ* fusion on the replicative vector pTCV-*lac* were grown in medium supplemented with Kanamycin. β-galactosidase assays were carried out on samples taken at hourly intervals as indicated. (A) *pagA-lacZ* reporter strains grown in LB broth in air at 37°C. (B) *pagA-lacZ* reporter strains grown in R Media with 0.8% NaHCO_3_ under 5% CO_2_ at 37°C. (C) *atxA-lacZ* reporter strains grown in R Media with 0.8% NaHCO_3_ under 5% CO_2_ at 37°C. Symbols in all panels: -□- 34F2 cell growth; -○- 34F2ΔBAS2714-12 cell growth; -▪- 34F2 LacZ expression; -•- 34F2ΔBAS2714-12 LacZ expression.

Expression of *pagA*, encoding the PA subunit of anthrax toxin, was monitored in different growth conditions, simulating host and non-host environments, known to affect virulence gene expression. A *pagA-lacZ* reporter on the replicative vector pTCV-*lac* [25] was transformed into the parental, the ΔBAS2714-12 and ΔBAS4675-77 strains and used to monitor *pagA* expression levels through β–galactosidase activity. To replicate non-host conditions that result in low-level expression of toxin genes, the strains were grown in LB broth in air under standard laboratory conditions (Figure 2A) while growth in defined R-medium in the presence of 0.8% NaHCO_3_ in a 5% atmosphere was used to mimic the host environment (Figure 2B). Deletion of the BAS4675-77 genes did not affect *pagA* expression in either growth condition tested indicating that this transport system did not have a role in bicarbonate transport and/or regulation of toxin gene expression and therefore was not further analyzed (data not shown).

The deletion of the BAS2714-12 genes did not affect *pagA* expression when cells were grown in LB in air suggesting that this system does not contribute to toxin expression under non-host growth conditions (Figure 2A). In contrast, when the strains were grown in defined R-medium under conditions known to induce toxin expression (0.8% NaHCO_3_ and 5% CO_2_), induction of *pagA* in the BAS2714-12 deletion strain was abolished compared to the parental strain (Figure 2B). These observations suggested that BAS2714-12 is required for induction of toxin expression under CO_2_/bicarbonate growth conditions believed to mimic the mammalian host.

The primary regulatory protein of toxin gene expression in *B. anthracis*, AtxA, is required for the observed induction of toxin expression in response to CO_2_/bicarbonate [18],[19]. Previous studies demonstrated that transcription of *atxA* is not directly induced in response to elevated CO_2_/bicarbonate [16]. To investigate the contribution of BAS2714-12 to *atxA* transcriptional regulation, an *atxA-lacZ* reporter carried on the pTCV-*lac* vector was electroporated in the 34F2 and 34F2ΔBAS2714-12 strains. Under the growth conditions that induced toxin expression and under which we observed a substantial difference in *pagA* expression, *atxA* expression was unchanged in 34F2ΔBAS2714-12 relative to the parental strain (Figure 2C). Thus, consistent with the lack of effect on *atxA* by the growth in the presence of CO_2_/bicarbonate [16], disruption of bicarbonate metabolism through deletion of the putative bicarbonate transporter BAS2714-12 did not affect *atxA* transcription.

To ensure that deletion of BAS2714-12 was responsible for the observed phenotypes, the BAS2714-12 deletion strain was complemented with these genes carried on a replicative plasmid. The BAS2714-12 locus, as well as a region 640 base pairs upstream of BAS2714 that may carry potential promoter and regulatory sequences, was cloned in the multicopy vector pHT315 to generate plasmid pAW144, and both plasmids were electroporated into strain 34F2ΔBAS2714-12. Expression of protective antigen was monitored by Western blotting on culture supernatants (Figure 3). When grown under toxin-inducing conditions, 34F2 supernatant samples contained detectable amounts of PA while 34F2ΔBAS2714-12 supernatant samples did not contain detectable levels of PA. When carrying the empty plasmid pHT315, PA remained undetectable in supernatant samples of the BAS2714-12 mutant strain while the presence of pAW144 restored PA expression, demonstrating that deletion of BAS2714-12 was, in fact, responsible for the elimination of toxin induction.

**Figure 3:** Western blotting using α-PA antibody. Strains grown in R Media with 0.8% NaHCO_3_ under 5% CO_2_ at 37°C supplemented with Erythromycin and Lincomycin as appropriate. Amount of sample loaded on 10% SDS-PAGE gel was normalized relative to cell density. Lane 1, MagicMark XP; Lane 2, 34F2 strain; Lane 3, 34F2ΔBAS2714-12 strain; Lane 4, 34F2ΔBAS2714-12 strain carrying plasmid pHT315; Lane 5, 34F2ΔBAS2714-12 strain carrying plasmid pAW144.

### Deletion of BAS2714-12 reduced bicarbonate uptake

The sequence similarity to known bicarbonate transporters and the elimination of bicarbonate-induced toxin expression following deletion suggested that BAS2714-12 may function as a bicarbonate transporter. To directly test the function of BAS2714-12 in bicarbonate transport, we compared the uptake of radiolabeled NaH^14^CO_3_ in the parental and mutant strain. Strains 34F2 and 34F2ΔBAS2714-12 were grown in R-media without added NaHCO_3_ in the presence of 5% CO_2_ to an OD_600_ of 0.4. NaH^14^CO_3_ was added to each culture, and uptake of NaH^14^CO_3_ was measured at several time points by liquid scintillation counting (Figure 4). The uptake of ^14^C in the 34F2ΔBAS2714-12 strain occurred at a significantly lower rate (6 fold) than in the parental 34F2 strain, indicative of disruption of bicarbonate uptake and providing further evidence that BAS2714-12 functions as a bicarbonate transporter.

**Figure 4:** Uptake of H^14^CO_3_^−^ by *B. anthracis* 34F2 and 34F2ΔBAS2714-12. Cells were grown in R Media without added NaHCO_3_ under 5% CO_2_ at 37°C to OD_600_ = 0.4. NaH^14^CO_3_ was added at time 0 and cell samples collected at times indicated. H^14^CO_3_^−^ uptake was determined by ^14^C accumulation in cells as measured by liquid scintillation counting; -▪- parental 34F2 strain, -•- 34F2ΔBAS2714-12 strain. Data was obtained from 3 independent cultures and error bars represent standard deviation from the mean.

### Carbonic anhydrase inhibitors do not significantly affect bicarbonate induction of toxin expression

Bicarbonate transporters import membrane-impermeable bicarbonate while carbonic anhydrase enzymes interconvert bicarbonate and CO_2_ and, thus, are able to convert membrane-permeable CO_2_ to bicarbonate [20]. Induction of toxin expression in *B. anthracis* is influenced by both bicarbonate and CO_2_, and, given the interconversion between the two compounds, separation of the relative influence of each compound on virulence has been difficult. The identification and deletion of the bicarbonate transporter essential to toxin induction now provided a tool to further probe the mechanism of induction.

A panel of available carbonic anhydrase inhibitors was tested including acetazolamide, ethoxyzolamide, hydrochlorothiazide and topiramate. Hydrochlorothiazide was found most efficacious as measured by reduced toxin expression levels (data not shown). In the presence of NaHCO_3_ and CO_2_, expression of *pagA-lacZ* in the parental strain 34F2 was identical with or without hydrochlorothiazide (Figure 5A). However, the residual *pagA-lacZ* expression in strain 34F2▵BAS2714-12 was completely inhibited by hydrochlorothiazide. Without added NaHCO_3_ but in the presence of atmospheric 5% CO_2_, hydrochlorothiazide reduced the expression of *pagA-lacZ* in the parental strain 34F2 and hydrochlorothiazide further reduced the level of *pagA-lacZ* expression in the 34F2ΔBAS2714-12 strain (Figure 5B). These data suggest that the residual *pagA-lacZ* expression in the absence of added NaHCO_3_ is due to the conversion of CO_2_ to ^−^HCO_3_ by carbonic anhydrase. These data also reinforce the concept that it is bicarbonate, and not CO_2_, that directly signals induction of virulence factor expression under host growth conditions.

**Figure 5:** Toxin gene expression in *B. anthracis* 34F2 and 34F2ΔBAS2714-12 in the presence of the carbonic anhydrase inhibitor hydrochlorothiazide. Cells carrying a *pagA-lacZ* fusion on the replicative vector pTCV-*lac* or promoter-less pTCV-*lac* were grown in medium supplemented with Kanamycin. β-galactosidase assays were carried out on samples taken at hourly intervals as indicated. (A) Strains grown in R Media with 0.8% NaHCO_3_ under 5% CO_2_ at 37°C. (B) Strains grown in R Media without added NaHCO_3_ under 5% CO_2_ at 37°C. Symbols in all panels: -▪- 34F2 *pagA-lacZ* expression; -□- 34F2 *pagA-lacZ* expression with 900 µM hydrochlorothiazide; -•- 34F2ΔBAS2714-12 *pagA-lacZ* expression; -○- 34F2ΔBAS2714-12 *pagA-lacZ* expression with 900 µM hydrochlorothiazide; -▴- 34F2 promoter-less pTCV-*lac* expression; -▵- 34F2 promoter-less pTCV-*lac* expression with 900 µM hydrochlorothiazide.

### Deletion of BAS2714-12 rendered *B. anthracis* avirulent in a mouse model of infection

While the role of CO_2_/bicarbonate in the induction of virulence gene expression is well demonstrated in laboratory batch cultures (*ex vivo*), no evidence has been provided yet that this role also is relevant in *B. anthracis* cells growing in the infected host (*in vivo*). In order to investigate whether the inability to import bicarbonate had any effect on the virulence of *B. anthracis*, an animal model of infection was used that employs a mouse strain highly susceptible to the unencapsulated Sterne strains [26]. Six week old female mice of the complement deficient strain A/J (The Jackson Laboratory) were injected subcutaneously with 10^6^ spores of the parental strain 34F2 or the 34F2▵BAS2714-12 mutant strain and monitored over the course of 12 days. A group of five A/J mice were infected for each strain. Within 54 hours, a mouse in the 34F2 control group infected with the parental strain showed significant swelling and reduced physical activity. Death occurred within the following 10 hours. In this group, two other mice became symptomatic and died within 72 hours, a fourth after 84 hours and the fifth mouse after 96 hours from the infection (Figure 6). In contrast, all 5 mice in the group infected with the mutant survived up to 12 days with no obvious signs of swelling or disease. While the parental strain is fully virulent in this mouse model, the ΔBAS2714-12 is avirulent, demonstrating for the first time that bicarbonate transport is essential to *B. anthracis* pathogenesis *in vivo*.

**Figure 6:** 34F2 and 34F2ΔBAS2714-12 in a mouse model of infection. A total of 10 6-week-old female A/J mice, 5 for 34F2 (-•-) and 5 for 34F2ΔBAS2714-12 (-▪-), were subcutaneously injected with 10^6^ spores and monitored over the course of 12 days. Mice were visually monitored daily for activity, and data expressed as percentage of survival.

## Discussion

*B. anthracis* must integrate numerous environmental signals to effectively replicate and induce disease. *B. anthracis* relies on a multiphasic lifestyle: non-metabolically active spores are necessary for infection and spread between hosts but are themselves incapable of replication while the metabolically active vegetative cells replicate and cause disease in the host but are incapable of dissemination between hosts. During the course of an infectious cycle, the pathways leading either to development through sporulation or to pathogenesis through toxin and capsule production are mutually exclusive suggesting the existence of a regulatory balance between the two pathways [27]. What the bacterium recognizes in the host as signals to induce pathogenesis mechanisms and the nature of the mechanisms necessary for commitment to development or pathogenesis remain poorly understood. Herein, we have identified an essential component for the induction of virulence gene expression in response to host bicarbonate levels and have exploited this finding to understand the extracellular and intracellular signals controlling virulence.

Our data demonstrated that the BAS2714-12 genes encode a previously uncharacterized bicarbonate ABC transporter. Similar ABC transporters have been identified and characterized in photosynthetic bacteria [21], but this is the first report of an ABC transporter involved in virulence in a pathogenic bacterial species. The BAS2714-12 system was originally annotated (Gen Bank: AE017225) as a putative sulfonate transporter, largely due to similarity to the characterized Ssu ABC transporter in *B. subtilis*. However, given the conservation between bicarbonate, nitrate, and sulfonate ABC transporters, the lack of characterized bicarbonate transporters in Gram-positive bacteria, and the difficulty in predicting the function of ABC transporters based upon nucleotide sequence, assignment of substrate specificity is ambiguous. Here we have shown that the ABC transporter encoded by BAS2714-12 is required for internalization of ^14^C-labeled bicarbonate. Together with the observation that the addition of taurine, a substrate of the *B. subtilis* Ssu system [28] and a commonly available sulfonate compound in the host, does not affect toxin gene expression and does not compete with bicarbonate induction (unpublished data) argues for the BAS2714-12 system as being specific for bicarbonate transport. The additional observation that the deletion of the BAS2714-12 genes eliminated the bicarbonate-dependent induction of toxin gene expression confirms a role for this transporter system in bicarbonate metabolism in *B. anthracis*.

Deletion of BAS2714-12 eliminates bicarbonate induction of *pagA* expression in growth conditions that mimic the animal host environment but does not significantly alter expression under non-inducing conditions. In LB media without added bicarbonate or CO_2_, conditions which mimic non-host and non-toxin inducing conditions, *pagA* expression is unaltered in the deletion strain. In contrast, when grown in R-media with added bicarbonate and CO_2_, conditions which mimic host and toxin inducing conditions, *pagA* expression remains very low in the mutant strain while *pagA* expression is strongly induced in the parental strain. These observations suggest that basal levels of *pagA* expression are unaffected by BAS2714-12 deletion, but, instead, the specific induction by bicarbonate requires the presence of BAS2714-12. Despite the strong effect of the BAS2714-12 deletion on toxin induction, the deletion strain shows no difference in growth under any condition tested relative to the parental strain, suggesting bicarbonate uptake through BAS2714-12 does not significantly contribute to non-virulence metabolic pathways under laboratory growth conditions. The deletion of BAS2714-12 can be complemented by supplying the locus *in trans* on a replicative plasmid. Small differences in *pagA* expression between the parental and deletion-complementation strains are likely due to differences in expression or gene copy number of BAS2714-12 carried on a relatively high copy number plasmid (15 copies/cell [29]).

The presence of the AtxA regulator is required for high-level expression of *pagA* in response to CO_2_/bicarbonate, but transcription of *atxA* is not directly regulated by CO_2_/bicarbonate [16]. Consistent with these observations, deletion of BAS2714-12 did not affect *atxA* transcription (Figure 2C).

The effect of BAS2714-12 on virulence in an *in vivo* animal model is drastic: while, as expected, infection of A/J mice with spores of the parental 34F2 strain quickly resulted in extensive edema followed by death [30], the infection with spores of the deletion strain showed no visual signs of infection and all mice survived to the end of the experiment (Figure 6). These results confirmed a correlation between the bicarbonate-dependent induction of toxin gene expression *ex vivo* and the virulence of *B. anthracis in vivo*. The A/J mouse model of infection was selected due to sensitivity to infection with the toxin-producing Sterne strain 34F2 (pXO1^+^ pXO2^−^). However, virulence in human hosts requires expression of both the toxin and the capsule. Capsule expression, like toxin production, is induced by bicarbonate [15]. Given the similar dependence of bicarbonate-induced capsule induction on both AtxA and genomic sequences [10],[15], it is likely that a BAS2714-12 deletion would abolish also the induction of capsule production and thus the virulence of a fully virulent, toxin- and capsule-producing strain.

Bicarbonate, and not CO_2_, appears to be the primary molecule regulating induction of virulence gene expression. If CO_2_ were the primary signaling molecule, one would expect a reduction of toxin expression in the presence of the carbonic anhydrase inhibitor as bicarbonate in solution can no longer be quickly converted into CO_2_ inside the cell. Instead, we observed the opposite phenomenon: inhibition of carbonic anhydrase activity only affects toxin expression in the absence of added bicarbonate or when bicarbonate can no longer be imported into the cell (Figure 5), conditions under which carbonic anhydrase would convert CO_2_ into bicarbonate. Induction of toxin expression *ex vivo* by high atmospheric CO_2_ levels in the absence of added bicarbonate is likely the result of spontaneous or carbonic anhydrase-driven conversion of CO_2_ into bicarbonate which then signals an increase in toxin expression. The sensor or metabolic pathway that directly responds to bicarbonate and induces toxin gene expression remains unknown, but its identification is an ongoing focus of our work.

Bicarbonate is a major element in the mammalian body. It is present in all body fluids and organs and plays a major role in acid-base homeostasis. The normal concentration of bicarbonate in the blood ranges between 22–26 mM and its presence, together with carbonic acid (H_2_CO_3_), hydrogen ions and carbon dioxide forms the buffering system required to provide resistance to drastic changes in pH values. Bicarbonate released from the pancreas also acts to regulate the pH in the small intestine to neutralize the acid entering the duodenum from the stomach [31],[32]. Thus bicarbonate may be a virulence signaling molecule for enterobacteria pathogenesis as well as blood borne pathogens.

*B. anthracis* is not alone among bacteria in regulating virulence gene expression in response to CO_2_/bicarbonate. CO_2_ and/or bicarbonate increases toxin production in *Vibrio cholerae* [33] and *Staphylococcus aureus* [34], induces expression of attachment genes in *Escherichia coli* O157:H7 [35], alters the antigenic profile of *Borrelia burgdorferi* [36], and activates a virulence regulatory protein in *Citrobacter rodentium* [37]. In any of these systems, a bicarbonate transport system similar to BAS2714-12 may be directly involved in bicarbonate transport and stimulation of virulence factor expression. Most directly relevant to bicarbonate regulation in *B. anthracis* is the stimulation of the antiphagocytotic M protein in *Streptococcus pyogenes* [38]. M protein expression is controlled by the regulatory protein Mga, a transcription factor that is similar to the *B. anthracis* AtxA regulatory protein, because it contains two PRD domains and may be subject to regulation by phosphorylation/dephosphorylation through the PTS carbohydrate utilization system [12],[39]. The apparent overlap of CO_2_/bicarbonate metabolic systems and regulation of PRD domains in regulatory proteins in response to carbohydrate utilization invites speculation of similar bicarbonate transport and regulatory systems between these pathogenic species. Interestingly, a BLAST search of the *S. pyogenes* M6 strain (Accession number NC_006086) using the BAS2713 substrate binding protein as query, identified the product of the Spy1045 gene as the protein with the strongest similarity (21%) and a TauA domain in its amino terminal half of the protein. In the C-terminal portion, Spy1045 contains an ABC-type permease domain (Binding-Protein-dependent transport system inner membrane component superfamily cl00427) that, together with the ATPase domain encoded by the Spy1046 gene (35% identity to BAS2714) may constitute the bicarbonate transporter of *S. pyogenes* (Figure 1).

The regulation of *B. anthracis* virulence factor requires a complex interaction between overlapping metabolic systems, but, for the first time, we have unraveled the dedicated transport components of the CO_2_/bicarbonate regulatory pathway. This has allowed us to directly separate the influences of multiple signaling molecules to discover that bicarbonate is directly responsible for the *in vivo* as well as *ex vivo* induction of virulence factor expression that is essential to *B. anthracis* pathogenesis. Notably, the availability of the 3-dimensional structure of the bicarbonate binding domain of the *Synechococcus* CmpA protein in the presence and absence of ligand may be exploited to uncover specific inhibitors of this domain and provide new avenues for antibacterial intervention [23]. In light of these findings, investigation of bicarbonate regulation and transport should be of much greater significance to a large number of pathogenic organisms.

## Materials and Methods

### Bacterial strains and growth conditions

*B. anthracis* Sterne 34F2 (pXO1^+^ pXO2^−^) and its derivatives were routinely grown in LB broth supplemented with the appropriate antibiotics at the following concentrations: chloramphenicol 7.5 µg/ml, tetracycline 5 µg/ml, erythromycin 5 µg/ml, lincomycin 25 µg/ml, or kanamycin 7.5 µg/ml. 5-bromo-4-chloro-3-indolyl-β-D-galactopyranoside (X-Gal) was added at a final concentration of 40 µg/ml to LB agar to monitor β-galactosidase activity in solid media. All carbonic anhydrase inhibitors (Sigma) were freshly prepared in DMSO immediately before addition to cultures. To induce high-level toxin expression, *B. anthracis* was grown in LB-agar plates or LB liquid media containing 0.8% sodium bicarbonate and 100 mM 4-(2-hydroxyethyl)-1-piperazineethanesulfonic acid (HEPES) [pH 8.0] or in R-Media [40] under 5% CO_2_. Electrocompetent *B. anthracis* cells were prepared following the method of Koehler *et al* [18].

The *E. coli* TG1 strain was used for plasmid construction and propagation. *E. coli* strain SCS110 was used for the production of unmethylated DNA for transformation in *B. anthracis*. *E. coli* transformation was performed by electroporation using the Bio-Rad Gene Pulser according to the supplier. Transformants were selected on LB broth supplemented with ampicillin (100 µg/ml), chloramphenicol (7.5 µg/ml), or kanamycin (30 µg/ml).

### Markerless gene deletion

Gene deletions in *B. anthracis* were generated essentially by the method of Janes and Stibitz [41]. A 738 bp region upstream of BAS2714 was amplified using primers BAS2714U5'Bam and BAS2714U3'Sal (Table S1) while an 828 bp region downstream of the BAS2712 was amplified using primers BAS2712D5'Sal and BAS2712D3'Pst. The sequenced products were then cloned into the temperature sensitive plasmid pORI-I-SceI [42] to generate plasmid pAW091. For deletion of BAS4675-77, a 624 bp region upstream of BAS4675 was amplified using primers BAS4675U5'Bam and BAS4675U3'Sal while a 750 bp region downstream of the BAS4677 was amplified using primers BAS4677D5'Sal and BAS4677D5'Pst. The sequenced products were also cloned in plasmid pORI-I-SceI to generate plasmid pAW093. Plasmids pAW091 and pAW093 were electroporated into *B. anthracis* 34F2 and grown at the permissive temperature of 28°C in the presence of chloramphenicol. Bacteria were then shifted to the non-permissive temperature of 37°C in the presence of chloramphenicol to achieve targeted plasmid integration by homologous recombination. Following plasmid integration, the protocol of Janes and Stibitz [41] was followed to generate the markerless deletion. Diagnostic PCR was carried out to ensure that the entire coding sequence had been correctly deleted. Diagnostic PCR was also carried out on genomic DNA using *atxA*-specific primers to ensure that the pXO1 plasmid was not lost during the process (Table S1).

### Complementation analysis

The BAS2714-12 region, including a region 640 base pairs upstream of BAS2714 containing potential regulatory sequences, was amplified using primers BAS27145'Xba and BAS27123'Hind and introduced into the pCR4Blunt-TOPO vector (Invitrogen). Following sequencing, the insert was removed by XbaI - HindIII digestion and ligated into XbaI – HindIII digested pHT315 multicopy plasmid vector [29], generating plasmid pAW144. pAW144, as well as pHT315 vector plasmid, was electroporated into both parental 34F2 and 34F2ΔBAS2714-12 strains. Diagnostic PCR was carried out on genomic DNA using *atxA* specific primers to ensure that the pXO1 plasmid was not lost during the process.

### β-Galactosidase assays

*B. anthracis* strains harboring the *pagA-lacZ* [12] or *atxA-lacZ* (pAtxA12 [17]) fusions on the replicative transcriptional fusion vector pTCV-lac [25] were grown at 37°C in LB or R medium supplemented with the appropriate antibiotics. β-galactosidase activity was assayed as described previously and specific activity was expressed in Miller units [43],[44].

### SDS-PAGE and Western blotting

*B. anthracis* strains were grown in R Media to approximately OD_600_ 1.0 for 8 hours in 5% CO_2_ atmosphere at 37°C, and supernatant samples were isolated by microcentrifugation of cell suspensions. SDS sample buffer was added to each supernatant, and samples were boiled for 5 minutes and loaded on 10% SDS-PAGE gels. The amount loaded was normalized relative to cell density. The gels were run at 30 mA for approximately 2 hr. The gels were transferred to a PVDF membrane (BioRad) in transfer buffer (25 mM Tris base, 192 mM glycine, 20% methanol) at 20 V overnight. The membranes were incubated for 30 minutes at room temperature in blocking buffer (5% dried milk in TBST (20 mM Tris-HCl pH 7.5, 150 mM NaCl, 0.1% Tween 20)) followed by addition of a polyclonal protective antigen antibody diluted 1∶10,000. The blots were washed 5 times and then incubated for 1 hour at room temperature with horseradish peroxidase-conjugated goat anti-rabbit antibody (BioRad) diluted 1∶10,000 in blocking buffer. Following washing of the membrane, binding of the antibodies was probed using the ECL Plus kit (GE) and the protein bands were visualized by PhosphorImager (Molecular Dynamics).

### Bicarbonate uptake analysis

Overnight cultures of *B. anthracis* 34F2 and 34F2ΔBAS2714-12 strains were diluted 1∶100 in R Media without added NaHCO_3_ and grown in 60 ml sterile culture bottles at 37°C in 5% CO_2_ atmosphere. When cultures reached an OD_600_ of 0.4, 50 µCi of NaH^14^CO_3_ (MP Biomedical) was added to each culture. At time intervals indicated, cells were separated from 1 ml of culture by vacuum filtration onto glass filters (Millipore) and immediately washed in 10 ml of cold medium. The filters were then placed in glass vials containing 5 ml of Bio-Safe II counting cocktail (RPI corp.), and radioactivity retained on the filter was measured in a Packard 1600 TR Liquid Scintillation Analyzer.

### Spore preparation

*B. anthracis* 34F2 and 34F2ΔBAS2714-12 strains were grown in Schaeffer's sporulation medium for approximately 72 hours until over 80% of spores were single and free by phase-contrast microscopy. Cells were collected by centrifugation at 10,000 g for 30 minutes, the medium was aspirated, and cell pellets resuspended in 20 ml of sterile distilled water. The cells were washed twice daily for 5 days by centrifugation at 12,000 g and resuspension in 20 ml fresh, sterile water in order to eliminate most vegetative cells. The cell pellets were then resuspended in 20% renografin (Squibb) and carefully layered over 50% renografin in a 30 ml Corex centrifuge tube. Tubes were then centrifuged at 13,000 g for 30 minutes. The supernatant containing vegetative forms was removed and the purified spore pellets were resuspended in 1 ml of sterile water. The spore pellets were washed twice daily for 3 days by microcentrifugation at 14,000 RPM followed by resuspension of spore pellet in 1 ml sterile water. Total spore counts were measured using a hemacytometer while live spore counts were measure by serial dilution followed by plating on LB-agar.

### Mouse infection

6-week-old female A/J mice (The Jackson Laboratory) were injected subcutaneously with 10^6^ renografin-purified spores. Progression of disease was monitored visually over 12 days. All mice were housed and maintained at The Scripps Research Institute animal facility under the approval of the Institutional Animal Care and Use Committee.

## Supporting Information

Table S1 Oligonucleotide primers used in this study
(0.04 MB PDF)
